# Analysis of Early Warning Diagnostic Indexes and Influencing Factors of Anxiety and Depression in Patients with Arrhythmia

**DOI:** 10.1155/2022/2061340

**Published:** 2022-10-15

**Authors:** Hao Yu, Yan Zhao, Yawen Li

**Affiliations:** Department of Cardiology, The Central Hospital of Dalian, Dalian, China

## Abstract

**Objective:**

Arrhythmia patients complicated with psychological problems are very common in clinics. The imbalance of autonomic nervous regulation of the heart caused by anxiety and depression will further promote the occurrence and development of arrhythmia. For nonorganic heart disease, *β* receptor blockers combined with antianxiety drugs have a good effect. Therefore, it is necessary to analyze the influencing factors of anxiety and depression in patients with arrhythmias.

**Methods:**

We included 150 patients with arrhythmia and divided them into observation groups (80 patients with anxiety and depression) and control groups (70 patients without anxiety and depression). All patients were monitored by Holter, and the detection of arrhythmia was compared between the two groups. We took the general situation and quality of life of the investigated patients as independent variables and the anxiety and depression status of the patients as dependent variables.

**Results:**

The detection rates of atrioventricular premature beats, ventricular premature beats, atrial fibrillation, short bursts of atrial tachycardia, and atrioventricular block in the observation group were all higher than those in the control group by dynamic electrocardiogram. Multivariate logistic stepwise regression analysis showed that age, years of education, obsessive-compulsive score, somatization score and alcohol consumption were the main influencing factors for anxiety and depression.

**Conclusions:**

The detection rate of arrhythmia in patients with anxiety/depression status was higher than in those without abnormal psychophylaxis. We should need to pay close attention to the risk factors of age, education years, obsessive-compulsive score, somatization score, and alcohol consumption, so as to prevent and timely detect anxiety and depression symptoms in patients with arrhythmias.

## 1. Introduction

Arrhythmia refers to any abnormality in the origin of cardiac impulses, heartbeat frequency, and rhythm, and impulse conduction. It can be caused by various organic cardiovascular diseases, drug poisoning, electrolyte and acid-base imbalance, and some arrhythmias can also be caused by autonomic nerve dysfunction [1, 2]. Arrhythmia complicated with anxiety or depression is very common in clinic. The latest data shows that the incidence of depression and anxiety among outpatients with arrhythmia is 20–30% [3]. The incidence in hospitalized patients can reach 40–60%. Anxiety and depression can activate hypothalamus-pituitary-adrenal system, promote sympathetic hypertonia, affect the coordination of autonomic nerves on cardiac regulation, and lead to the occurrence or aggravation of arrhythmia [4]. Research shows that both organic heart disease and nonorganic heart disease patients will produce obvious anxiety and depression symptoms, which will further aggravate the occurrence and development of arrhythmias and even lead to an increase in the mortality of organic heart disease patients [5, 6].

Anxiety in the field of psychology often refers to an inner uneasiness or groundless fear aroused by the lack of obvious and objective reasons [7, 8]. In fact, it does not happen in reality, but it is a kind of nervous, worried, and fearful emotion caused by my expectation that I will face bad or even dangerous situations. It is mainly manifested as continuous tension, uneasiness, worry, accompanied by mental tension, restlessness, excessive small movements, and excessive emotion and crying, and even panics [9]. At the same time, most patients will also be complicated with symptoms of autonomic nervous dysfunction such as chest tightness, dry mouth, palpitation, tremors of both hands, cold sweat, anorexia, and constipation [10]. Contrary to the common people's understanding, an appropriate sense of anxiety will not bring negative effects to mankind, but rather the positive factors of human life can provide positive life motivation [11]. However, excessive anxiety will have a significant negative impact on people, not only as a manifestation of mental illness but also when accompanied by physical illness. If the heart rate accelerates and the blood pressure rises, and then the ventricular fibrillation threshold are lowered, the risk of sudden death from coronary heart disease is greatly increased [12]. Similar to anxiety, depression is also a common bad mood, which refers to the mental state dominated by a low mood. It often occurs together with bad emotions such as anxiety, helplessness, and agitation, and physical discomfort such as insomnia. There are various causes of depression, but only about 35% of depressed patients are caused by simple stress events, and about 65% of patients are related to somatic diseases [13]. Some studies have confirmed that depression can cause cortisol hyperfunction, improve sympathetic sensitivity, increase the corresponding hormone level in plasma, and then, cause insulin resistance, pancreatic islet secretion defect, lipid metabolism disorder, and other endocrine disorders, increase the incidence of obesity, and further aggravate the severity of arrhythmia [14, 15].

The prognosis of arrhythmia is related to the etiology, inducement, evolution trend and whether it leads to serious hemodynamic disorder [16]. It can suddenly attack and cause sudden death, and can also continue to involve the heart and cause failure. The poor prognosis and sudden death rate of cardiovascular diseases are increasing, which are related to bad psychology, disease cognition, and emotional reactions, especially anxiety and depression [17]. Emotions play an important role in the occurrence, development, and outcome of arrhythmia patients, especially the common bad emotions such as anxiety and depression [18]. Therefore, the identification and diagnosis of anxiety and depression disorders are directly related to the therapeutic effect and prognosis of arrhythmias [19].

Anxiety and depression can induce and promote arrhythmias in patients with cardiovascular diseases, and Holter can effectively reflect the relationship between them. Holter is one of the most convenient methods for arrhythmia detection and evaluation [20]. Various arrhythmias can be detected by Holter. Holter is a method that can continuously record and compile ECG changes of the human heart in an active and quiet state for a long time [21]. This technology was first applied to the study of monitoring cardiac electrical activity by Holter in 1947, so it is also called the Holter monitoring electrocardiograph, and it has become one of the important diagnostic methods of nontraumatic examination in the clinical cardiovascular field. Compared with ordinary ECG, Holter can continuously record up to 100,000 ECG signals within 24 hours, which can improve the detection rate of nonsustained arrhythmias, especially transient arrhythmias and transient myocardial ischemia attacks [22]. Holter is widely used, mainly for capturing paroxysmal arrhythmias, such as paroxysmal tachycardia and premature beats, and recording their occurrence time, quantity, and distribution; whether there is transient angina pectoris, myocardial ischemia, and the inducement and time of attack. Anxiety and depression patients often seek medical treatment for cardiovascular symptoms such as palpitation, chest tightness, fatigue, etc. ventricular or atrial arrhythmia often occurs in 24 h Holter [23]. Depression and anxiety can lead to a series of physiological and pathological changes by causing dysfunction of autonomic nervous system and enhancement of sympathetic nerve activity in vivo, thus, increasing the activity of catecholamine system, thus, inducing coronary artery spasm, exacerbating myocardial ischemia, and causing the formation of abnormal autonomy of the original nonautonomic cardiomyocytes under the effect of excessive catecholamine secretion [24]. The release of procoagulant substances and angiotensin II makes the sympathetic nerve excited, the heart rate accelerates, the blood pressure increases, the perceptual domain decreases, the HRV decreases, and the QT dispersion increases, which leads to an increase in cardiac load and a decrease in the threshold of ventricular ectopic activation, thus causing malignant ventricular arrhythmias with poor prognosis [25]. The comparison of the detection rates of arrhythmias in anxiety and depression patients by Holter ECG showed that the detection rates of atrial premature beats, ventricular premature beats, and short bursts of atrial tachycardia, atrial fibrillation, and atrioventricular block were significantly increased [26]. Therefore, Holter may be used as an early diagnosis and an early warning index of anxiety and depression in patients with arrhythmia.

With the rapid development of social economy, fast-paced lifestyle, social loneliness, excessive Internet use, overeating, or excessive dieting, as well as various life stress events have caused huge psychological and physiological burdens, of which anxiety and depression accompanied by arrhythmias are the most common [27, 28]. The novelty of this study was to detect the rate of arrhythmia in patients with anxiety status was higher than those without abnormal psychophylaxis.

## 2. Materials and Methods

We consecutively included 150 patients hospitalized in our hospital due to arrhythmia from January 2021 to April 2022 in our hospital. Inclusion criteria: Meeting the diagnostic criteria of arrhythmia; all have basic reading and writing ability and clear consciousness. Exclusion criteria: Patients with physical or mental diseases other than feelings of anxiety and depression; history of cardiac intervention and surgery; blind and deaf; pregnant or lactating women. There were 134 males and 16 females. The average age was (46.43 ± 5.12) years old. Disease types were as follows: 88 cases of paroxysmal supraventricular tachycardia, 30 cases of preexcitation syndrome, 18 cases of frequent ventricular premature beats, and 14 cases of atrial fibrillation. The study was approved by the ethics committee of our hospital, and all patients signed informed consent.

General information of all selected patients, including treatment mode, life behavior, body mass index, hospitalization time before treatment. Anxiety and depression were assessed by self-assessment of depression and self-assessment of anxiety. Both self-assessment of depression and self-assessment of anxiety had 20 self-assessment items. The higher the score, the higher the degree of anxiety and depression. The median value was 40 points. The Self-rating Depression Scale (SDS) and Self-rating Anxiety Scale (SAS) questionnaires were used to assess the anxiety and depression of the patients. If the SDS score was ≥50, the patients would be assessed as depresssion, and if the SAS score was ≥50, the patients would be assessed as anxiety. The patients' self-assessment and the professional doctors of our hospital would conduct blind assessment. The quality of life was investigated with the Chinese version of Symptom Checklist 90 (SCL-90) scale. The 70 items included in the scale can be summarized into 7 symptom groups, including somatization Compulsion, interpersonal sensitivity, hostility, terror, paranoia, psychosis. The higher the score, the worse the quality of life.

All patients were monitored by Holter monitoring (CV3000 12 lead Holter recording and analysis system, Beijing gushanfeng company). Holter was recorded continuously for 24 hours. The occurrence of arrhythmia was determined manually and automatically by computer system. The detection of arrhythmia in the two groups was statistically analyzed. The influencing factors of anxiety and depression in patients with arrhythmia were investigated and analyzed by professionals according to the above three scales. The evaluation was completed within 15–20 minutes. The questionnaire was collected and checked on-site to ensure that the effective rate of the survey was 100%.

### 2.1. Statistical Analysis

SPSS 25.00 statistical software was used, *t*-test was used for measurement data, and (%) was used for counting data *χ*2 inspection. For multiple comparisons, data were analyzed via analysis of variance (ANOVA) with the Tukey–Kramer multiple comparisons test. The influencing factors were analyzed by dichotomous logistic stepwise regression, and *P* < 0.05 means that the difference is statistically significant.

## 3. Results

### 3.1. Baseline Demographic Data

The smoking rate of the patients in the observation group was higher and the number of years of education decreased was lower than that of the control group (*P* < 0.05), but there were no statistical difference in alcohol consumption, disease course, body mass index (BMI), and hospitalization time (*P* > 0.05) (Table 1).

### 3.2. The Type of Arrhythmia in Patients with/without Anxiety and Depression Status

The detection rates of atrial premature beats, ventricular premature beats, and short bursts of atrial tachycardia, atrial fibrillation, and atrioventricular block in the observation group were significantly higher than those in the control group. Data analysis found that the difference was statistically significant (*P* < 0.05, Table 2).

### 3.3. The Quality of Life Scores of the Two Groups

The scores of somatization, compulsion, interpersonal sensitivity, hostility, terror, paranoia and psychosis in the observation group were significantly increased (*P* < 0.05), which are shown in Table 3.

Binary logistic stepwise regression analysis of the influencing factors of anxiety and depression in patients with arrhythmia.

We took the general situation and quality of life from the survey as independent variables and the anxiety and depression status of the patients as dependent variables, and included them in the binary logistic stepwise regression analysis. The results showed that age, years of education, obsessive-compulsive score, somatization score, and alcohol consumption were the main influencing factors leading to anxiety and depression (*P* < 0.05), which are shown in Table 4.

## 4. Discussion

The most common arrhythmia is premature cardiac beats, including atrial premature beats and ventricular premature beats. Patients often have chest tightness, palpitations, heartbeat or shortness of breath, and an individual cough. Premature beats often occur in patients with nonorganic heart disease, and are often related to mental tension, excitement, drinking, strong tea, and coffee [29]. Through 24-hour ECG dynamic monitoring, it was found that the incidence of premature contraction in nervous workers was twice as high as that in general workers. Palpitation, chest tightness, and other symptoms of patients with premature beats are not necessarily related to premature beats but can also be caused by anxiety and depression. Anxiety and depression can also increase the incidence of premature beats [30]. When premature beats are combined with anxiety and depression, the activation of the hypothalamus-pituitary adrenal system, the promotion of sympathetic hypertonia, and the release of too many catecholamines lead to abnormal myocardial autonomy and the posterior depolarization of increased Ca influx, thus leading to an increase in the incidence of premature beats [31]. In this study, 150 patients with premature cardiac beats were scored by the Hamilton scale, which showed that all the included cases were accompanied by obvious anxiety and depression. All patients were randomly divided into antianxiety and depression treatment group and the control group. The results showed that the incidence of premature cardiac beats in the fluocinonide treatment group was significantly reduced compared with the control group, and the cardiac-related symptoms were also significantly reduced. Arrhythmias associated with common nonorganic heart diseases include idiopathic ventricular tachycardia, idiopathic atrial fibrillation, atrial flutter, and atrial tachycardia. The symptoms of chest tightness and palpitation are more obvious during the attack, and because the attacks are repeated and without any incentive, patients are often more prone to anxiety and depression. Premature beats, atrial fibrillation, ventricular tachycardia, ventricular fibrillation, conduction block and other arrhythmias can occur in various heart diseases, such as coronary heart disease, hypertension, heart failure, cardiomyopathy and so on. The occurrence of arrhythmias often predicts the aggravation of the original heart diseases, makes the conditions and symptoms more complex and diverse, and aggravates the anxiety or depression of patients. This change of mood can further accelerate the deterioration of the disease [32]. Studies have shown that arrhythmia patients with anxiety and depression have more serious dysfunction of the autonomic nerve in regulating the heart, which usually leads to increased sympathetic activity and decreased parasympathetic activity [33, 34]. A large number of studies have shown that the prevalence of anxiety in patients with coronary heart disease is as high as 40%∼70%. When depression and anxiety occur in patients with coronary heart disease, it can cause a large amount of catecholamines to be secreted in the body, leading to an accelerated heart rate [35]. Studies have shown that anxiety and depression in patients with coronary heart disease can not only increase the incidence of arrhythmia but also greatly increase mortality. A very important factor in the pathophysiological mechanism of chronic heart failure is the activation of the renin-angiotensin-aldosterone system, which in turn aggravates the process of heart failure. Moreover, it is easy to promote rapid ventricular arrhythmia, and anxiety and depression will promote the activation of sympathetic nerves, which will further aggravate heart failure and increase the incidence of malignant arrhythmia and sudden death in patients with chronic heart failure [36].

Electrocardiograms are often used to monitor patients with cardiovascular diseases, which have different characteristics at different periods of time [37]. Through dynamic electrocardiogram monitoring, it was found that the detection rate of arrhythmia accompanied by anxiety and depression in the observation group was significantly higher than that in the control group, and the difference was statistically significant (*P* < 0.05), suggesting that anxiety and depression were closely related to the occurrence of arrhythmia. This study believes that anxiety and depression can trigger autonomic nervous disorders in the body and further increase the cardiac load with the release of procoagulant substances and angiotensin II, reducing the threshold of ventricular ectopic activation and triggering malignant ventricular arrhythmia. Arrhythmia is complicated by anxiety and depression, which is closely related to arrhythmia. The detection rate of arrhythmia in patients monitored by Holter is high, which has clinical application value.

Anxiety and depression are common mental disorders in the clinic. Studies have shown that anxiety and depression are common psychological disorders in patients undergoing interventional treatment, and about 6.0% of patients suffer from anxiety and depression symptoms. The results showed that the education level, regional distribution, marital status, and nature of work of patients with arteriosclerosis were related to their accompanying emotional disorders. The level of the patient's education determines a person's ability to acquire knowledge and broaden their vision to another level. Because of their remote families, rural patients are inconvenient to seek medical treatment, and their economic conditions are generally worse than those of urban patients, with large emotional fluctuations. Moreover, rural patients have more contact with their neighbors and friends and are more susceptible to the attitude of the surrounding people. For those with a high educational level, for various reasons, they often sit for a long time, exercise less, stay up late, smoke and drink too much for entertainment, or surf the Internet too much, which will lead to obesity, endocrine disorders, immune system disorders, and other harmful cardiovascular and cerebrovascular elasticity [38]. People with low education generally engage in more physical labor, relatively more exercise, good spirits, reduced physical pressure, and less vascular damage. At the same time, exercise is conducive to emotional relief. Therefore, people with low education have a higher rate of arteriosclerosis than those with high education, especially those with mental skills. Those who have social support, especially those who have family members and caregivers, will have a less psychological burden than those who are alone. Even if they are ill, because their families accompany and support them, their morale is relatively stable.

If these influencing factors were given timely and appropriate health education, the prevention of primary diseases could be effectively improved. Health education shall be given to medical staff and inpatients, and targeted health education shall be given to different types of arteriosclerosis diseases. We should widely publicize the knowledge about psychological snow and arteriosclerosis, explain to patients or their families the importance of long-term exercise and health care, pay attention to weight control, and adhere to a low salt and low fat diet; pay attention to emotional adjustment and keep a happy mind; stick to physical exercise. At the same time, it is necessary to explain the general knowledge of psychology and general physical diseases, especially arteriosclerosis, to the patients' families in a targeted way, so that the families can have a general understanding of the diagnosis and treatment of the disease, support and care for the patients. On the other hand, patients should constantly learn, understand themselves, adapt to the environment, control their emotions, vent appropriately, and reduce psychological pressure. People who worry about and fear diseases should know that these are controllable diseases, and they should persist in taking drugs when necessary. When side effects of drugs occur, they can be identified and dealt with in time, so as to avoid aggravating side effects and causing greater pain and affecting patients' emotions [38].

Antianxiety and depression treatment is effective and meaningful in both chronic diseases and acute stress events. Therefore, in the prevention of anxiety and depression, health education, purpose, related complications, and other information are conveyed to patients, and targeted psychological intervention is carried out for patients, which can significantly improve their psychological coping ability and promote their physical and mental recovery. The limitation of the study was that the number of patients is not so large. Also, the mechanism was not clarified. Further studies are needed to study the mechanism.

In conclusion, the detection rate of arrhythmias in elderly patients with cardiovascular disease combined with anxiety and depression under Holter monitoring is high, and anxiety and depression are closely related to the occurrence of arrhythmias in elderly patients with cardiovascular disease. We need to pay close attention to the risk factors of age, education years, obsessive-compulsive rating, somatization rating, and alcohol consumption so as to prevent and timely detect anxiety and depression in patients with arrhythmias.

## Figures and Tables

**Table 1:** Baseline demographic characteristics.

Index	Observation group	Control group	*P*-value
Age (years)	55.43 ± 5.53	48.26 ± 6.75	0.015^*∗*^
Drinking (*n*)	21 (26.25)	7 (10.00)	0.012^*∗*^
Smoking (*n*)	17 (21.25)	15 (20.14)	0.925
Course of disease (months)	4.33 ± 1.30	4.39 ± 0.97	0.202
Years of education (years)	9.20 ± 4.31	14.29 ± 4.24	0.015^*∗*^
Body mass index (BMI, kg/m^2^)	21.76 ± 4.11	21.76 ± 4.18	0.313
Hospitalization time (days)	14.44 ± 0.67	14.40 ± 0.66	0.472

**Table 2:** Type of arrhythmia in patients with/without anxiety and depression status.

Type	Observation group	Control group	*P* value
Atrioventricular premature beats	48 (60.00)	21 (30.00)	0.006
Ventricular premature beats	32 (40.00)	13 (18.57)	0.003
Atrial tachycardia	21 (26.25)	7 (10.00)	0.002
Atrial fibrillation	17 (21.25)	5 (7.14)	0.005
Atrioventricular block	13 (16.25)	2 (2.86)	0.012

**Table 3:** The quality-of-life scores in patients with/without anxiety and depression status.

Index	Observation group	Control group	*P -value*
Somatization	1.65 ± 0.45	1.38 ± 0.41	0.010
Forced scoring	1.55 ± 0.59	1.46 ± 0.42	0.013
Sensitivity to human nature	1.50 ± 0.44	1.34 ± 0.35	0.016
Hostile	1.54 ± 0.47	1.32 ± 0.33	0.018
Terror	1.69 ± 0.51	1.50 ± 0.36	0.019
Paranoia	1.49 ± 0.35	1.36 ± 0.34	0.025
Psychosis score	1.35 ± 0.31	1.22 ± 0.22	0.028

**Table 4:** Analysis of the influencing factors of anxiety and depression in patients with arrhythmia.

Variable	*B-value*	*P value*	*OR-value*
Age	1.398	0.013	5.231
Years of education	1.690	0.004	4.872
Forced scoring	1.701	0.006	4.982
Somatization score	1.600	0.015	0.203
Drinking	1.573	0.007	0.502

## Data Availability

The data used to support this study are available from the corresponding author upon request.
